The article "Diagnosis of Blood Vessel Stenosis Caused by Arterial Thrombosis of Lower Extremities by Ultrasound Based on the Mobile Information System" was retracted in 2022. Reason: compromised peer review.

# Diagnosis of Blood Vessel Stenosis Caused by Arterial Thrombosis of Lower Extremities by Ultrasound Based on the Mobile Information System

**DOI:** 10.1155/2022/7282192

**Published:** 2022-02-26

**Authors:** Lianfeng Wu, Chenchen Zhang

**Affiliations:** Color Ultrasonic Room, Jinan Municipal Hospital of Traditional Chinese Medicine, Jinan 250012, Shandong, China

## Abstract

The thrombosis process is a multifactorial evolution process that includes many genetic and environmental factors that interact with each other. It refers to the existence of blood deposits in the heart or blood vessel walls or abnormal blood clots in the circulatory blood flow during the survival period of humans or animals for some reason. This article aims to analyze the research of blood vessel stenosis caused by arterial thrombosis of the lower extremities under the diagnosis of cardiac ultrasound based on the mobile information system. This article first introduces the mobile information nursing system and its development process. The mobile nursing information system has experienced three stages of development and is an important application of the further development of science and technology in medical information technology. It also proposes a medical diagnosis method based on SRM on a mobile platform and gives a technical roadmap for heart sound analysis and processing. Then, based on the mobile information system, the formation of arterial thrombosis in the lower extremities was analyzed and discussed in the ultrasound diagnosis of the heart, and the vascular stenosis caused by the arterial thrombosis of the lower extremities was analyzed by imaging. Experimental results show that when there is >50% stenosis or complete occlusion, the CTA false positive is more prominent, especially when the calf artery type is complete stenosis. The main cause is that the circulation of the lower limbs is very poor, the blood entering the blood vessels of the lower limbs is scarce, the capillaries are weakly enhanced, and the quality cannot be improved.

## 1. Introduction

Due to the significant improvement in the lives of the majority of people in recent years, human dietary composition and changes in habits have gradually undergone great changes. In addition, factors such as the aging of people and the reduction of infectious diseases have caused the incidence of various vascular diseases to increase, and they have become the primary diseases that threaten human physical and mental health and even life. Arteriosclerosis occlusion and thrombosis in some important parts are some of the most common initiating factors for the main clinical symptoms of these diseases. Among them, acute arterial thrombosis (AT) is gradually formed in the arterial stenosis segment, and to a certain extent, there is the formation of collateral circulation. The onset is less sudden and the condition is alleviated. The etiology includes rupture of atherosclerotic plaque and induced thrombus formation at the rupture site, low flow state (congestive heart failure, hypovolemia, hypotension, etc.), hypercoagulable state, aortic dissection, or lower extremity arterial dissection.

At present, it is believed that the pathogenesis of arterial thrombotic diseases is very complicated, including genetic influence, environment, age, gender, smoking, atherosclerosis, and hypertension. Many reasons can promote the formation and development of arterial thrombosis. Further clarification of the formation mechanism of arterial thrombosis will provide a theoretical basis for preventing the formation of arterial thrombosis and even reversing the process of thrombosis. It has made a significant contribution to medicine in the prevention of arterial thrombosis and vascular stenosis.

According to the research progress at home and abroad, different scholars also have a certain degree of cooperation in the field of cardiac ultrasound diagnosis, lower extremity arterial thrombosis, and mobile information systems: Marantz P proposed a predictive model based on echocardiographic results to estimate the possibility that CHD fetuses need neonatal cardiac invasive treatment, including cardiac surgery or catheter treatment. The prediction model based on the results of CHD fetal echocardiography can accurately estimate the possibility of neonatal cardiac invasive treatment even if there is no clear diagnosis. This may change patient care, especially in areas where there are no fetal medicine specialists or pediatric cardiologists, and referrals can be extremely difficult due to social and economic barriers [1]. In recent years, great progress has been made in the use of lung ultrasound to detect edema and interstitial changes in the lungs. Soldati G. aims to describe the latest knowledge about the response of the pleural plane to ultrasound to explore the difference between ultrasound-related interstitial syndromes related to lung disease and ultrasound related to cardiogenic edema [2]. Gonzalez-Hadad A. uses ultrasound as the main screening tool for finding occult heart injuries and found that ultrasound has a sensitivity of 79% and a specificity of 92% in the diagnosis of occult penetrating heart wounds. However, it should be used with caution in patients with heart injury and left hemothorax at the same time [3]. Patients with peripheral arterial disease (PAD) have an increased risk of acute limb ischemia (Ali), which is mainly caused by thromboembolic disease in atherosclerotic plaque or proximal emboli. Irani Z. introduced four Ali patients. In these patients, EPD was used during intra-arterial thrombolytic infusion, thereby reducing dissolution time and pain, while retaining the distal runoff blood vessels [4]. Puz P. aims to study carotid artery stenosis that can lead to brain tissue damage and microembolism complications related to intracranial arterial blood flow disorders. The results show that the microembolic signal in patients with symptomatic carotid artery stenosis is one of the ultrasonic features of unstable carotid artery stenosis, and the worse reactivity parameters of cerebral arteries are related to severe carotid artery stenosis [5]. Jones RS reported on the design and manufacture of a three-dimensional (3D) in vitro system to simulate vascular stenosis so that specific cell interactions and responses to hemodynamic stimuli can be studied. Tubular cellularization constructs (cell tubes) are produced using a collagen molding system to create a stenotic artery model [6]. Filho I. aims to provide a case study of the deformation process in the mobile application development process based on the existing Web information system and introduced the design and execution of a case study to investigate the feasibility of using the metamorphosis process to create mobile applications based on existing Web information systems [7]. However, these scholars did not analyze the causes of vascular stenosis caused by thrombosis of the lower extremities under the diagnosis of cardiac ultrasound based on the mobile information system but only unilaterally explored their significance.

The innovations of this paper are mainly reflected in the following. (1) First, it introduces the mobile information nursing system and its development process, proposes a method of medical diagnosis based on the mobile platform of SRM, and gives a technical roadmap for heart sound analysis and processing. (2) Then, based on the mobile information system, the formation of arterial thrombosis in the lower extremities was analyzed and discussed in the ultrasound diagnosis of the heart, and the vascular stenosis caused by the formation of arterial thrombosis in the lower extremities was analyzed by imaging.

## 2. Method Based on the Mobile Information System in the Cardiac Ultrasound Diagnosis of Vascular Stenosis Caused by Lower Extremity Arterial Thrombosis

### 2.1. Mobile Information Nursing System

The nursing information system is an information system that uses information technology, computer technology, and network communication technology to collect, store, process, transmit, and query nursing management and business technical information to improve the quality of nursing management. It is an important subsystem of the hospital information system. With the widespread application of computers in the medical field, information technology has gradually penetrated into the nursing field, and the emergence of nursing information systems has its inevitability. With the widespread application of computers in the medical field, information technology has gradually penetrated into the nursing field, and the emergence of nursing information systems has its inevitability. The mobile communication system is a kind of radio communication system, which mainly includes a cellular system, a trunking system, an Ad Hoc network system, a satellite communication system, a packet wireless network, a cordless telephone system, and a radio paging system. Among them, the nursing information system has the characteristics of a wide range of sources, a wide range of sources, a wide range of sources, and a large amount of randomness. Among them, mobile medicine is to provide medical services and information through the use of mobile communication technologies such as PDAs, mobile phones, and satellite communications. In particular, in the field of mobile Internet, it is mainly based on medical and health App applications based on mobile terminal systems such as Android and iOS. Mobile medical care has changed the traditional way of life that people could only go to the hospital to “see a doctor” in the past. Whether at home or on the road, people can always listen to the advice of doctors or obtain various health-related pieces of information. Mobile medical care can help improve the problem of seeing a doctor. Since the launch of the new medical reform, the demand and development potential of China's medical and health industry informatization are huge, accelerate the advancement of the medical and health information business, and deepen the medical and health industry to become the focus of the industry.

The nurse information system has gone through several years of research and development. It can also be said that it has experienced three stages of development. These three stages have witnessed the development history of the nurse information system and are also an important application of the further development of science and technology in medical information technology. These three stages are the manual nurse stage, professional nurse information system stage, and mobile nurse information system [8].

The first stage is the manual nursing stage, but this stage can also be said to be not a complete nursing system, or an independent nursing system, with only the standard text of nurses, nurse processes, and some nurse record files [9]. Nursing staff carry out clinical nursing in accordance with nurse record specifications, manuals, etc., after the completion of the nurse's work, prepare nurse documents, including temperature sheets, nurse record sheets, and other nurse documents, and finally file and seal the paper nurse documents [10]. This stage consumes huge manpower and material resources, so nursing work can also be said to be a completely manual method [11].  Figure 1 shows the working care environment based on the mobile information system. In the later stage of this stage, a nurse station management system was produced, which is a management system that interacts with the medical care management system and centrally manages the patient information system. In this system, nursing-related information management is rarely involved [12]. In this system, some doctors can also print the patient's infusion worksheet and then paste it on the infusion bottle to verify the infusion work drug list and patient information with the nursing staff. However, these verification methods are only manual methods. In busy nurse work, the nurse staff must be cautious, which will increase the work pressure of the nurses virtually [13].

The second stage is to produce a special nurse system to assist nursing staff to go to work. All medical records, nurse files, etc. have electronic files, so nurses do not have to fill in paper data files [14]. In this way, patient care information is easy to store and read. There are two document recording methods at this stage: one is to save the nursing record in the form of text; another feature is that the personal care files stored in a structured method are stored in a structured method. Compared with the file format, the structured preservation method has greater value superiority [15]. In data statistics and biomedical research, data analysis can be used to maintain patient information security. Compared with the traditional nursing stage, this stage has great advantages [16]. However, this stage did not reduce the work of nursing staff, nor did it improve the quality of nurses' service. Nursing staff still have to finish nursing work at the bedside and return to the nurse workstation to complete nursing records on the computer [17]. For patient checks, drug checks can only be done manually, so this stage is not supported by the majority of nursing staff, but this stage lays a good foundation for the next stage and is an important part of the development of nursing informatization [18].  Figure 2 is a system architecture diagram based on mobile information nursing.

The third stage is the mobile nursing information system. This stage is based on the previous stage and introduces the concept of mobility. Through the introduction of mobile facilities, all nurse records and nurse papers can be realized at the bedside. At the same time, the mobile facilities can also realize the verification of information, so as to record the actual nursing time. The progress of this stage depends on the progress of wireless network technology, mobile devices, Internet of Things technology, and computer systems. At present, there have been various degrees of research on mobile nursing at home and abroad, and some achievements have also been made [19].

### 2.2. SRM-Based Mobile Platform Medical Diagnosis Method

SRM method is a new method for state analysis and evaluation, which belongs to the category of pattern recognition. This method was first applied to the monitoring of bridge health structure and achieved good results. In order to extend the SRM method to medical signal processing, such as cell image recognition, genetic analysis and evaluation, three-high data evaluation and analysis, and pathological slice analysis, the theoretical basis of the SRM method will be introduced below [20].

The concept of SRM is established from the following equation of motion:

(1) $$\begin{array}{c} F\alpha^{\prime \prime }+E\alpha^{\prime }+J\alpha =0. \end{array}$$

For a single degree of freedom system, it is easier to get the mass *F*, damping *E,* and stiffness *J*; then, the vibration frequency can be obtained.

(2) $$\begin{array}{c} s^{2}=\frac{J}{F}-\frac{E^{2}}{4F^{2}}. \end{array}$$

Then, there are

(3) $$\begin{array}{c} F=\frac{J\pm \sqrt{J^{2}-{\left(sE\right)}^{2}}}{2s^{2}}=y\left(J,s,E\right). \end{array}$$

For a multidegree-of-freedom system, it is very difficult to determine the parameters for the system, because the mass F, damping *E*, and stiffness *J* have a certain relationship with the structure of the system, so in fact, this problem is very complicated [21]. The multidegree-of-freedom system is generally expressed as ∑_*n*_*y*(*J*_*n*_, *s*_*n*_, *E*_*n*_)=*F*_total_, namely,

(4) $$\begin{array}{c} \sum_{n}\frac{1}{F_{\text{total}}}y\left(J_{n},s_{n},E_{n}\right)=1\left(\text{constant}\right). \end{array}$$

Using Taylor's formula, *y*(*J*_*n*_, *s*_*n*_, *E*_*n*_) can be extended to

(5) $$\begin{array}{c} \sum_{n}B_{n}\left(J_{n},E_{n}\right)s_{n}+u\left(s_{1},s_{2},\ldots ,s_{m}\right)=1. \end{array}$$

It can also be written as

(6) $$\begin{array}{c} \sum_{n}b_{n}s_{n}+u\left(s_{1},s_{2},\ldots ,s_{m}\right)=1. \end{array}$$

In the above formula, *b* : =(*b*_1_, *b*_2_,…, *b*_*m*_) is the structural parameter of the system and *s* : =(*s*_1_, *s*_2_,…, *s*_*m*_) is the response characteristic of the system. This formula can be written as

(7) $$\begin{array}{c} y\left(b,s\right)=1. \end{array}$$

*y*(*b*, *s*) is called the system state equation, and we use *β* to represent the system state later; then,

(8) $$\begin{array}{c} \beta =y\left(b,s\right). \end{array}$$

Any matter in the world can be regarded as a system. The state of the system depends on its own internal factors and external factors and is essentially determined by its own structure or structural attributes and the natural environment [22]. The SRM method can be used to define and record the state changes of a system. When the system does not change, *β* is a constant; namely,

(9) $$\begin{array}{c} \beta =y\left(b,s\right)\\ =1. \end{array}$$

In the linear model, the nonlinear part *s*(*s*_1_, *s*_2_,…, *s*_*m*_) is 0, and only the linear part on the left, namely, ∑_*n*_*b*_*n*_*s*_*n*_=1, is considered; then,

(10) $$\begin{array}{c} b=\frac{s}{s^{2}}. \end{array}$$

Because in general, a system will have multiple feature vectors from different perspectives, here is a weight for each vector:

(11) $$\begin{array}{c} \varphi_{n}\in \left[0,1\right],\\ \sum_{n=1}^{f}\varphi_{n}=1. \end{array}$$

Then, the structural parameter *b* of the system can be approximately written as

(12) $$\begin{array}{c} b=\sum_{n}^{f}\varphi_{n}\frac{s_{n}}{s^{2}}. \end{array}$$

Therefore, we express the system state in the linear model as

(13) $$\begin{array}{c} y\left(b,s\right)=\sum_{n}^{f}\varphi_{n}\frac{s_{n}}{s^{2}},s\\ =\sum_{n}^{f}\varphi_{n}\frac{s_{n}}{s^{2}},\frac{s}{s^{2}}. \end{array}$$

In a health monitoring system, we usually only get the status response feature, and the response feature matrix *s*(*s*_1_, *s*_2_,…, *s*_*m*_) can be obtained by using various feature extraction methods. Later, we use two other symbols *r* and *t* instead of *b* and *s* to represent the structural parameters and response characteristics of the system respectively [23]. It is transformed into the following state description equation to represent

(14) $$\begin{array}{c} \beta =y\left(r,t\right)\\ =1. \end{array}$$

In the above formula, *β* is the system state variable (the value is a fixed constant when the system has not changed), and *r* and *t*, respectively, correspond to the structural parameters and response characteristics of the system. Among them, *β* is the quantification of the dual relationship between *r* and *t* [24].

After uniform variables, the system state can be further expressed as

(15) $$\begin{array}{c} y\left(r,t\right)=\sum_{n}^{f}r_{n}l_{n},t, \end{array}$$

where *l*_*n*_=*s*_*n*_/‖*s*‖^2^ and *t*=*s*/‖*s*‖^2^.

Similar to the SVM method, the SRM method also cleverly uses the kernel function, which greatly simplifies the processing of high-dimensional feature vectors [25]. By using the kernel function, the above formula can be transformed into a nonlinear form:

(16) $$\begin{array}{c} \beta =y\left(r,t\right)\\ =\sum_{n}^{f}r_{n}j\left(l_{n},t\right). \end{array}$$

Of course, the reasonable use of the kernel function is also one of the key issues in the SRM method.  Figure 3 shows the perception model of the kernel function.

The kernel function can usually be selected by the following methods:

1. The existing expert experience is used to select the kernel function.
2. The cross-validation method is adopted, different kernel functions are used for experiments, and the kernel function with the smallest induction error is selected.
3. Using the hybrid kernel function method, compared with the above two methods, this method of selecting kernel function has become the current mainstream method. The research results prove that the combination of polynomial and Gaussian kernels can not only satisfy good learning ability but also achieve good generalization.

For all feature vectors *l*_*n*_ to be tested, there are

(17) $$\begin{array}{c} \beta =y\left(r,t\right)\\ =\sum_{n}^{f}r_{n}l_{n},t\\ =e. \end{array}$$

In the above formula, *l*_*n*_ and *t* are both related to the response characteristics of the system.

When there is no change in a system, the state equation of the system should be equal to a certain constant; namely,

(18) $$\begin{array}{c} \beta =y\left(r,t\right)\\ =\sum_{n}^{f}r_{n}j\left(l_{n},t\right)\\ =e. \end{array}$$

*f* in the formula represents the number of eigenvalues.

This article defines the kernel function:

(19) $$\begin{array}{c} j\left(u,t\right)=\text{exp}\left(-\frac{g\left(u,t\right)}{\varepsilon^{2}}\right). \end{array}$$

In the formula, the scale *ε* determines the sensitivity to the difference between two different states of the same system. The larger the scale, the less sensitive to system differences; that is, the degree of discrimination decreases. Conversely, the smaller the selected scale, the higher the sensitivity to system differences, and the higher the degree of discrimination. However, if the scale is too large or too small, distortion may be caused, and the specific scale value needs to be set according to the actual situation.

Now, we define a Gram-Schmidt matrix *D*:

(20) $$\begin{array}{c} D=\left[\begin{array}{c} j\left(h_{1},h_{1}\right),j\left(h_{1},h_{2}\right)\ldots j\left(h_{1},h_{n}\right)\\ j\left(h_{2},h_{1}\right),j\left(h_{2},h_{2}\right)\ldots j\left(h_{2},h_{n}\right)\\ \cdots \\ j\left(h_{n},h_{1}\right),j\left(h_{n},h_{2}\right)\ldots j\left(h_{n},h_{n}\right) \end{array}\right]. \end{array}$$

From (18), we can get

(21) $$\begin{array}{c} \left[\begin{array}{c} y\left(r,t_{1}\right)\\ y\left(r,t_{2}\right)\\ \cdots \\ y\left(r,t_{n}\right) \end{array}\right]=D\left[\begin{array}{c} r_{1}\\ r_{2}\\ \cdots \\ r_{n} \end{array}\right]\\ =\text{Dr}=\text{ev.} \end{array}$$

Then, there is Dr=ev=1/*n* *vv*^*I*^Dr; that is,

(22) $$\begin{array}{c} \left(Q-\frac{1}{n}\;vv^{I}\right)\text{Dr}=0. \end{array}$$

Find the least-squares solution of the above formula:

(23) $$\begin{array}{c} \text{min}\left(Q-\frac{1}{n}\;vv^{I}\right){\text{Dr}}^{2}. \end{array}$$

Notice *r*_*n*_ ∈ [0,1] and ∑_*n*=1_^*f*^*r*_*n*_=1.

The heart sound diagnosis system based on the mobile platform uses a new analysis method-SRM to classify and recognize heart sound signals. While expanding the application field of the SRM method, it also brings a new method route to the current heart health state detection. The combination of the SRM method and mobile platform technology has created a service software for smartphone users that can monitor their heartbeat at any time, which can save the cost of diagnosis and treatment for patients to a certain extent. But it also saves a lot of hospital resources and can reduce the morbidity and mortality of cardiovascular diseases to a great extent.  Figure 4 shows the technical roadmap of heart sound analysis and processing.

## 3. Experimental Results Based on the Mobile Information System in the Diagnosis of Vascular Stenosis Caused by Lower Extremity Arterial Thrombosis in Cardiac Ultrasound

### 3.1. Arterial Thrombosis of Lower Extremities Based on the Mobile Information System in Cardiac Ultrasound Diagnosis

The clinical symptoms of arterial thrombosis are pain, where the pain is often the first symptom, gradually extending to the distance; the skin color and temperature change; the blood circulation of the limbs being impaired; the skin being wax-like pale; arterial pulsation being weakened or disappeared; numbness; and dyskinesia. The winter preventive measures for arterial thrombosis include the following: keep warm; keep warm; tonic should be moderate. The patients with arterial thrombosis are mainly middle-aged and elderly people and people with high blood pressure, high blood fat, high (blood) viscosity, and high smoking addiction. There are people with coronary heart disease, people with myocardial infarction, people with atrial fibrillation, atherosclerosis, and people with abdominal aortic aneurysms. Venous thrombosis of the lower extremities is a common peripheral vascular disease. Venous valve insufficiency and concurrent pulmonary embolism caused by venous thrombosis of the lower extremities are a major danger to the patient's labor and life safety.

Among them, the ultrasound used for medical diagnosis is mainly pulse reflection technology, including A-type, B-type, D-type, M-type, and V-type. From the perspective of development trends, ultrasound has been progressing toward the color display and three-dimensional display. In addition, penetration technology and tissue characterization are also being studied by many ultrasound workers. Ultrasound diagnosis can be applied to acute inflammation, abscesses, cysts, effusions, stones, foreign bodies, tumors, trauma, and perforation of cavities and organs in various parts of tissues and organs.

Gender and age: there were 18 males and 12 females in the treatment group; the oldest was 70 years old and the younger was 30 years old; both were 59.14 ± 9.93 years old. In the control group, there were 16 males and 14 females; the oldest was 70 years old, and the youngest was 39 years old, all between 60.52 ± 7.79 years old. After statistical data processing, there is no significant difference between the two groups (*P* > 0.05), which is more reliable.

Among the 30 patients in this group, 6 cases had no clear cause; 8 cases were cured by surgery, including 1 case after debridement due to enlarged craniotomy due to epidural hematoma, one case after great saphenous varices, two cases after total internal hysterectomy, one case after splenic rupture, two cases after femoral hernia resection, and one case after radical resection of rectal cancer. Eleven patients were lying supine for a long time, including five patients who were paralyzed for a long time due to cerebral infarction, and two patients were fixed by plaster due to a fracture of the lower arm. Two cases were treated conservatively after spleen contusion and laceration caused by serious trauma such as a car accident, and two cases were accompanied by bedsores due to elderly patients. Two cases suffered cold due to long-term use of contraceptive measures or long-term outdoor work in the first half of five years. Among the 30 patients in the control group, 7 cases had no clear cause, there were 10 cases after surgical treatment, of which 3 cases were due to varicose great saphenous blood vessels, and 1 case was splenectomy due to severe abdominal trauma causing damage to the spleen. There were one case of postoperative treatment for tibiofibular fractures, two cases of total internal hysterectomy for uterine fibroids, one case after debridement due to burns of both lower limbs, one case after inguinal hernia surgery, and one case after huge liposarcoma resection due to lower limb movement. Twelve cases were bedridden for a long time, including two cases with soft cell contusion of the lower arm due to severe trauma and three cases with plaster or splint external fixation due to fractures. Four cases were bedridden for a long time due to acute cerebral infarction, one case was conservatively treated for renal contusion caused by severe trauma, two cases were conservatively treated for lumbar compression fractures, and one case was cold.

Lesion location and type of clinical diagnosis: in the patient group, there were 23 cases of left limb, 3 cases of right limb, and 4 cases of double limbs; the control group had 20 cases of left limb, 8 cases of right limb, and 2 cases of double limbs. The patient has a group of peripheral types with nine limbs, central type with seven limbs, and mixed type with eighteen limbs. In the control group, ten limbs were peripheral type, eight limbs were central type, and 14 limbs were mixed type.  Figure 5(a) is the analysis of the patient's lesion location, and Figure 5(b) is the analysis of the patient's clinical type.

Among the 30 patients in the treatment group, 7 cases were treated by clinical application, 12 cases were markedly effective, 8 cases were effective, and 3 cases failed. The overall effective rate was 90.00%.  Figure 6 shows the comparison of the total curative effect between the two groups of patients.

Before the diagnosis of the two groups of patients, the circumference change was very small, and there was no clear and significant difference (*P* > 0.05).  Figure 7(a) is a comparison of the patient's limb circumference difference.

The D-dimer concentration of the two groups of patients before treatment was basically the same, and there was no significant difference (*P* > 0.05).  Figure 7(b) shows the average D-dimer content of patients before treatment.

The total evaluation of arterial patency before the diagnosis of the two groups of patients was basically the same, and there was no significant difference (*P* > 0.05). The total evaluation of arterial patency in the diagnosis group and the control group decreased significantly after diagnosis than before diagnosis, and there was a significant difference between the two (*P* < 0.01).  Figure 8 shows the changes in arterial patency before and after treatment.

### 3.2. Imaging Analysis of Vascular Stenosis Caused by Arterial Thrombosis of the Lower Extremities

There are many reasons for cerebrovascular stenosis, and they are related to age. For example, the age of onset of vascular stenosis caused by nodular arteritis is usually 10 to 30 years old. However, people with atherosclerosis and stenosis are usually middle-aged and elderly people between 40 and 80 years old or even older people. Children who get sick are mostly caused by congenital abnormalities of vascular development. Cervical spondylosis is also a predisposing factor of cerebrovascular stenosis.

All patients had successfully done DST and CTA examinations. Except for one patient who had mild contrast allergy, no other major complications occurred. In addition, the performance of all patients' vascular reconstruction images is good, and the image quality can meet the treatment indicators. The diseases are roughly divided into the following three categories for comparison: (1) extra-iliac blood vessel type: the main lesions are in the iliac blood vessels, including the total skeletal blood vessels, as well as the internal and external skeletal blood vessels; (2) femoral artery type: the lesion is located in the femoral and rouge blood vessels; (3) calf blood vessel type: the lesion is mainly in the calf blood vessel, which is divided into anterior tibial, posterior, and drainage vessel types.  Table 1 shows the comparison of iliac artery type CTA and DSA.

Comparison of sensitivity, characteristic, and accuracy: the two are relatively compared. CTA is sensitive; characteristics and accuracy are reduced as the diseased blood vessel becomes thinner. The sensitivity, specificity, and accuracy of CTA are 95%, 88%, and 90%, respectively.  Table 2 shows the comparison of femoral and popliteal DSA and CTA.

Comparison of collateral circulatory system: the performance of the collateral circulatory system, due to the narrowing of the tumor diseased blood vessels, compared with CTA and DSA, is getting worse and worse. In DSA imaging, for patients with significantly poorer collateral circulatory system, the results of reimaging after increasing the amount of contrast reagent and increasing the exposure time indicate that the visibility of the distal capillaries and collateral circulatory system of the occluded lesion can be improved.  Table 3 shows the comparison between DSA and CTA of calf arterial type.  Table 4 shows the comparison of conventional and increased-dose time-lapse imaging of lower extremity arterial occlusion lesions.

The image characteristics of chronic coronary atherosclerosis stenosis of the limbs in DSA angiography: coronary atherosclerosis of the limbs is usually narrow, but the whole area is narrow, as shown in Figures 9 and 10. Since the blood in the upper and lower arms is relatively slow, when the vascular stenosis rate reaches 93%, it is easy to cause the blood supply to be interrupted and secondary thrombosis, and a rat tail or blind end appears at the end of a completely closed blood vessel. If accompanied by thrombosis, a cup sign appears. Due to the long course of lower arm atherosclerotic stenosis, obviously thickened collateral vessels can often be seen.

Most patients with peripheral vascular stenosis occlusive disease initially manifest as intermittent trekking, but as the disease progresses, resting state pain caused by ischemia or necrosis, long-term nonhealing ulcers, infection, and gangrene will gradually occur in the future. In this case, stents and high-current surgery can repair and improve the blood circulation of the limbs; otherwise, it will cause amputation. Therefore, after completing the basic physical and ultrasound tests, the main tasks of angiography are to determine the scope of the disease, evaluate the severity of the disease, evaluate the distant blood circulation, and determine the unpredictable new disease. According to the early clinical manifestations of peripheral vascular stenosis and occlusive disease, according to the location, size, severity, and multiple or single diseases of stenosis and occlusive disease, and according to the general condition of the patient, the specific diagnosis method was determined.

## 4. Discussion

In the results of this survey, when the stenosis is less than 50%, the difference between DSA and CTA is generally in mild stenosis. The reasons are as follows. (1) There are human reasons when the doctor measures the capillary caliber of the lesion. (2) It is related to the direct scanning inspection technology: the difference between DSA and CTA is poor in spatial resolution, and the difference caused by the thickness of the layer can be directly scanned. When there is >50% stenosis or complete occlusion, CTA false positive is prominent, especially when the calf artery is completely stenosis. The reasons are as follows. (1) In some patients with poor limb circulatory systems, the contrast agent entering into the limb capillary is very small, the capillary enhancement is very weak, and the quality is difficult to guarantee. (2) Because the scanning time and the peak time of the intravascular control agent are highly required, too early or too late will cause errors in the intravascular performance, and the peak time of detecting the target capillary will be biased. (3) Insufficient estimation of the control agent: due to the lack of the content of the control agent, it cannot meet the density values of different reconstructions, resulting in deviations. But with the discovery and use of 64-layer and more CT, this aspect will be improved and strengthened. Most patients with peripheral vascular stenosis occlusive disease initially manifest as intermittent trekking, but as the disease progresses, resting state pain caused by ischemia or necrosis, long-term nonhealing ulcers, infection, and gangrene will gradually occur in the future. In this case, stents and high-current surgery can repair and improve the blood circulation of the limbs; otherwise, it will cause amputation.

## 5. Conclusions

DVT refers to a thrombus formed by abnormal accumulation of blood components such as platelets, fibrinogen, and human red blood cells in the arterial capillary lumen. DVT is more common in clinical medicine, but in recent years, with the changes in the human diet and living habits, fatty diets and sedentary phenomena have gradually increased. As a result, the blood has always maintained a hypercoagulable state, so the incidence of DVT is gradually increasing. However, if the early detection of DVT disease cannot be carried out, or the early and reasonable treatment is carried out, it can lead to chronic deep artery valve dysfunction and have a certain impact on the patient's working environment and quality of life. Until there is a significant disability and a significant reduction in the quality of life, it is of great significance to explore more effective treatment methods. However, modern medical research points out that the three biggest causes of DVT are capillary wall damage, blood stagnation, and plasma hypercoagulability and have basically formed a clinical consensus. Arterial thrombosis of the lower extremities is a common clinical peripheral thrombosis. Its occurrence is rapid, and if the thrombus falls off, it can cause fatal pulmonary embolism, which is life-threatening. Due to time and funding constraints, the sample size of this study is relatively small. Therefore, the next step of research still needs to set up multiple randomized, prospective, large-sample, and multicenter clinical trials to increase the credibility and scientificity of the research. In addition, it is necessary to further study the deep-seated action mechanism and specific action links of the prescription.

## Figures and Tables

**Figure 1:** Work nursing environment based on the mobile information system.

**Figure 2:** System architecture diagram.

**Figure 3:** The kernel function perception model.

**Figure 4:** The technical route of heart sound analysis and processing.

**Figure 5:** Analysis of the location and clinical types of patients.

**Figure 6:** Comparison of the total curative effect between the two groups of patients and the total score of TCM syndromes.

**Figure 7:** Comparison of the patient's limb circumference difference and the patient's D-dimer content before and after treatment.

**Figure 8:** Changes in the fibrinogen content and arterial patency rate before and after treatment.

**Figure 9:** Arteriosclerosis and stenosis of the lower extremities.

**Figure 10:** Image in DSA.

**Table 1:** Comparison of iliac artery types CTA and DSA.

Parameter	DSA	CTA	*P* value
Arterial clarity	3.8	3.9	*P* > 0.05
Lumen stenosis	43	45	*P* > 0.05
Sensitivity	100%	95%	*P* > 0.05
Characteristic	100%	88%	*P* > 0.05
Accuracy	100%	89%	*P* > 0.05
Lateral branch circulation	Display well	Display well	—

**Table 2:** Comparison of femoral and popliteal artery types DSA and CTA.

Parameter	DSA	CTA	*P* value
Arterial clarity	3.5	3.7	*P* > 0.05
Lumen stenosis	80	45	*P* > 0.05
Sensitivity	100%	93%	*P* > 0.05
Characteristic	100%	83%	*P* > 0.05
Accuracy	100%	90%	*P* > 0.05
Lateral branch circulation	Display well	Display general	-

**Table 3:** Comparison of calf arterial DSA and CTA.

Parameter	DSA	CTA	*P* value
Arterial clarity	3.6	3.2	*P* > 0.05
Lumen stenosis	49	49	*P* > 0.05
Sensitivity	100%	96%	*P* > 0.05
Characteristic	100%	87%	*P* > 0.05
Accuracy	100%	83%	*P* > 0.05
Lateral branch circulation	Display general	Display poor	-

**Table 4:** Comparison of conventional and increased-dose time-lapse imaging of lower extremity arterial occlusion lesions.

	Iliac artery type		Femoral and popliteal artery type		Calf arterial type	
	Conventional	Increase	Conventional	Increase	Conventional	Increase
Dose	9	16	16	18	15	24
Lateral branch circulation	Clear	Clear	Light	Clear	Not clear	Clear
Distal vessel	Display	Clear	Light	Clear	Not clear	Display
Evaluation	Excellent	Excellent	Good	Excellent	Difference	Good

## Data Availability

No data were used to support this study.
